# lncRNA H19 Promotes Ox-LDL-Induced Dysfunction of Human Aortic Endothelial Cells through the miR-152/VEGFA Axis

**DOI:** 10.1155/2022/3795060

**Published:** 2022-03-19

**Authors:** Feng Tang, Siqi Zhang, Honghao Wang, Shijia Xu, Sen Yang, Xiaohan Zhu, Huan Zeng, Yongyao Yang

**Affiliations:** ^1^Department of Cardiology, The Second People's Hospital of Guiyang, Guiyang 550023, China; ^2^College of Life Science, Zhejiang University, Hangzhou 310058, China; ^3^Department of Cardiology, Guizhou Provincial People's Hospital, Guiyang 550023, China

## Abstract

**Objective:**

lncRNA H19 (H19) elevation is related to the risk of coronary artery disease. DIANA-lncBase database analysis suggested that microRNA-152 (miR-152) and H19 have binding sites. Here, the effect and mechanism of H19 and miR-152 in the oxidized low-density lipoprotein (ox-LDL)-induced human aortic endothelial cells (HAECs) were explored.

**Methods:**

The expression of H19, miR-152, and vascular endothelial growth factor (VEGF)-A in the HAECs treated with 5 *μ*g/mL ox-LDL was detected by qRT-PCR. MTT, wound-healing assay, and tube formation assay were analyzed to evaluate the angiogenic activity of H19 and miR-152 in the HAECs cells knocked down H19. Dual-luciferase assay was performed to verify the targeting relationship of miR-152 to either H19 or VEGFA, respectively. Western blot was used to detect the expression of epithelial-mesenchymal transition (EMT)-related proteins (E-cadherin and vimentin) and VEGFA protein in the cells.

**Results:**

After ox-LDL treatment, the expression of H19 and VEGFA was significantly increased, miR-152 expression was remarkably decreased. H19 was mainly expressed in the cytoplasm of HAECs. Knocking down H19 or overexpression of miR-152 significantly inhibited the cellular proliferation, migration, tube formation, and EMT trend of the HAECs. On the contrary, miR-152 interference reversed H19 silencing-mediated effects in the ox-LDL-induced HAECs. The dual-luciferase assay showed that miR-152 had a targeting relationship with H19 and VEGFA. MiR-152 was negatively corrected with the VEGFA expression.

**Conclusion:**

Ox-LDL negatively regulates miR-152 via H19, promotes the expression of VEGFA, and induces the dysfunction of HAECs.

## 1. Introduction

Cardiovascular diseases (CVDs) are characterized by high morbidity and mortality, which seriously threaten global adults and constitute a major socioeconomic burden on global economic growth [1]. Atherosclerosis is the major underlying cause of CVDs. Atherosclerosis is a widespread chronic inflammatory disease of the arterial wall, which usually leads to disability or even death [2]. Previous studies have shown that the main mechanism of atherosclerosis is lipid accumulation and chronic inflammation in the arterial wall, while atherosclerosis is usually associated with altered lipid metabolism and hypercholesterolemia [3]. Oxidized low-density lipoprotein (ox-LDL) is a known risk factor for CVDs, which expresses the heterogeneous oxidative changes of the lipid portion of LDL and apolipoprotein B (ApoB) [4]. Studies have pointed out that plasma levels of ox-LDL in patients with atherosclerotic CVDs are elevated. Moreover, clinically, the level of the ox-LDL or anti-ox-LDL antibody is selected as a biomarker for predicting cardiovascular events [5]. Overproduction of ox-LDL leads to abnormal proliferation, apoptosis, migration, angiogenesis, and inflammatory responses, all of which are responsible for endothelial cell dysregulation [6]. It is suggested that ox-LDL can be used as a new therapeutic target for the treatment of atherosclerosis and cardiovascular diseases.

Epithelial-mesenchymal transition (EMT) plays a crucial role in progress and destabilizing atherosclerotic plaques via infiltration of fibroblasts and upregulation of matrix metalloproteinase [7, 8]. Downregulation of E-cadherin is a hallmark of EMT [9]. Abnormality of E-cadherin in foam cells during the process of atherosclerosis suggests that lipid accumulation may relate to the reorganization of cellular interactions in atherogenesis [10]. In the EMT process, vimentin maintains intracellular homeostasis via regulation of cytoskeleton architecture and cellular force generation [11]. Gong et al. [12] recently showed that vimentin promotes atherogenesis in ApoE^−/-^ mice. These data indicate that both E-cadherin and vimentin are important factors of EMT and have pathological activities in atherosclerosis.

lncRNA is a type of long-chain non-coding RNA larger than 200 nt. Early studies have confirmed that lncRNA can be used as a signal molecule to participate in cellular growth and development, as well as the occurrence and development of diseases [13]. Some studies have pointed out that lncRNA is an important information transmission mediator between cells and tissues, which can transmit information efficiently and accurately [14]. Studies have shown that lncRNA can promote tumor growth and metastasis. lncRNA MALAT1 can promote tumorigenesis through the Wnt/*β*-catenin pathway, EMT, phosphatidylinositol kinase (PI3K)/protein kinase B (AKT) pathway, extracellular regulatory protein kinase (ERK)/mitogen-activated protein kinase (MAPK) pathway, and angiogenesis [15]. lncRNA PCGEM1 is a specific lncRNA for prostate cancer, which can promote cell proliferation and reduce apoptosis induced by anticancer drugs [16]. A number of research have shown that the expression of lncRNA H19 (H19) in cancer cell lines and samples of patients with cancer is significantly upregulated [17]. After knocking down the H19, the viability, invasion, and migration ability of cancer cell lines were significantly reduced [18]. It shows that H19 has a great relationship with the biological activity of cells. Some studies reveal that increase of H19 is related to the risk of coronary artery disease [19]. Further, other scholars found that H19 is involved in the process of atherosclerosis. Sun et al. reported that knocking down the H19 can prevent atherosclerosis deterioration by increasing p53-mediated apoptosis in vascular smooth muscle cells [20]. Zhang et al. [21] revealed that knocking down H19 could regulate the proliferation and apoptosis of vascular smooth muscle cells induced by ox-LDL through the miR-148b/Wnt/*β*-catenin pathway. Thus, H19 is closely related to the formation of atherosclerosis and is an important mediator of the ox-LDL damaged vascular cells. At the same time, studies have found that H19 regulates the apoptosis of vascular endothelial cells in occlusive arteriosclerosis through the NF-*κ*B pathway [22]. However, no research has revealed the role of H19 in the process of ox-LDL inducing vascular endothelial cells. Therefore, in order to explore the effect of H19 on atherosclerosis, this study aims to elucidate the pathological mechanism of ox-LDL-induced vascular endothelial cell lesions *in vitro*, which would provide new therapeutic targets for atherosclerosis.

## 2. Materials and Methods

### 2.1. Cell Culture and Grouping

Human aortic endothelial cells (HAECs) were purchased from the American Type Culture Collection (ATCC; Manassas, VA, USA). The cells were cultured in complete Dulbecco's modified Eagle's medium (DMEM) (Gibco, Waltham, MA, USA) containing 10% fetal bovine serum (FBS) (Gibco), 100 mg/mL penicillin, and 100 mg/mL streptomycin (Gibco) at 37°C and 5% CO_2_ in an incubator (ThermoFisher Scientific, Waltham, MA, USA). Wild-type HAECs were used as negative controls (Control group). HAECs treated with 5 *μ*g/mL of ox-LDL [23] (Feather biology, Shanghai, China) for 24 h were used as the ox-LDL group. H19 siRNA (si-H19) and siRNA scramble (si-NC), miR-152 inhibitor and NC inhibitor, miR-152 mimics and mimics NC, vascular endothelial growth factor (VEGF)-A overexpression plasmids (VEGFA) were all designed and synthesized by Guangzhou Ruibo Biotech (Guangdong, China) and transfected with Lipofectamine 3000 (ThermoFisher) by following the manufacture instructions in the ox-LDL-treated HAECs.

### 2.2. Quantitative Real-Time Polymerase Chain Reaction (qRT-PCR)

The nucleus and cytoplasm of HAECs were isolated by a Subcellular Protein Fractionation Kit for Cultured Cells (ThermoFisher). Total RNA of the cells in each treatment group was extracted by TRIzol reagent (ThermoFisher) according to the instruction. The extracted RNA was detected by a NanoDrop microspectrophotometer (ThermoFisher), and cDNA was prepared according to the High-Capacity cDNA Reverse Transcription Kits (ThermoFisher). QRT-PCR analysis was performed according to the instructions of the SYBR GREEN kit (TaKaRa, Tokyo, Japan) to detect the expression levels of H19, miR-152, VEGFA mRNA, and other genes. Glyceraldehyde-3-phosphate dehydrogenase (GAPDH) was used as an internal reference control. Each experiment was set with 6 replicates. The experimental data obtained by qRT-PCR were calculated using the 2^−ΔΔCt^ method to calculate the relative expression of the target gene. The primer sequence is shown in Table 1.

### 2.3. Detection of Cellular Growth by Thiazolyl Blue (MTT) Staining

After treatment, each group of cells in the logarithmic growth phase was seeded in a 96-well plate at a density of 5000 cells/well, cultured in complete DMEM for 24, 48, and 72 h. 20 *μ*L of 5 mg/mL MTT (Sigma-Aldrich, St. Louis, MO, USA) solution was added into each well of the cells and incubated in a 37^o^C incubator for 4 h. Following this, the supernatant was discarded, 150 *μ*L of DMSO was added, and shaken for 15 minutes. The absorbance value of each well was measured with a wavelength of 570 nm in a microplate reader.

### 2.4. Wound-Healing Assay

Cells from each group were seeded into a 6-well plate, cultured to confluence. A 10 *μ*L sterile pipette tip was used to scratch the diameter vertical to the horizontal plane of a single well. Cell debris and detached cells were removed by washing with PBS. Fresh serum-free medium was added, cultured for 24 h, and photographs were taken with an inverted microscope to record the experimental results. ImageJ software was used to calculate the cellular migrated area on the scratched space. Each assay was repeated thrice.

### 2.5. Tube Formation Assay

100 *μ*L of Matrigel (HD Biosciences, San Diego, CA, USA) was added to each well of a 24-well plate and incubated at 37°C for 30 min. Cells treated with different conditions were resuspended in FBS-free DMEM and seeded at a concentration of 1 × 10^5^ cells/well. After 6 h, the formation of capillary structures was counted under a light microscope, and scanning and quantification were performed. Each assay was repeated thrice.

### 2.6. Double-Luciferase Reporter Gene Assay

The sequence of H19, miR-152, and VEGFA binding site and their mutant sequences were inserted into the downstream of the firefly luciferase gene to construct an expression vector (Promega, Madison, Wisconsin, USA). MiR-152 mimics/mimics NC and mammalian cell miRNA reporter plasmid pmirGLO (Qincheng Biotechnology, Shanghai, China)-H19-WT/MUT recombinant plasmid, miR-152 mimics/mimics NC and pmirGLO-VEGFA-WT/MUT, and recombinant plasmid and Lipo2000 liposomes were mixed, respectively, and transfected into 293T cells (ATCC). After transfection 48 h, luciferase activity was detected according to the instructions of the Dual Luciferase Reporter Gene Assay kit (Promega).

### 2.7. Western Blot

Detecting cells were lysed by an RIPA reagent (Beyotime Biotechnology, Shanghai, China) to extract total protein. The protein concentration of the lysates was detected with a BCA kit (Abcam, Cambridge, British). Each 20 *μ*g of the lysate protein was mixed with 4 x Protein Loading Buffer and boiled for denaturation, separated by SDS-PAGE, and was transferred on PVDF membranes. 5% skimmed milk was used to block the nonspecific proteins for 1 h. The primary antibody was reacted with the membrane overnight at 4°C. After washing, the membrane reacted with the secondary antibody for 1 h at room temperature. After washing, a chemiluminescence reagent (Haoxin-Biotech, Hanzhou, China) was applied to visualize the probed protein. The image was analyzed in an imaging system. Densitometry of the target protein bands was evaluated using ImageJ software, and the relative protein expression was calculated using *β*-actin as an internal reference.

### 2.8. Statistical Analysis

The tested results were analyzed by one-way ANOVA and independent samples *t-test* analysis with SPSS 26.0 (IBM-SPSS, Chicago, IL, USA). Results were expressed as mean ± standard deviation (SD). The correlation between miR-152 and H19/VEGFA was analyzed by the Pearson correlation analysis. *P* < 0.05 was used as the criterion for judging the significance of the difference.

## 3. Results

### 3.1. Ox-LDL Induced Upregulation of H19 Expression and Downregulation of miR-152 Expression in HAECs

DIANA-lncBase database (https://diana.e-ce.uth.gr/lncbasev3/interactions) predicted that miR-152 and H19 have binding sites (Figure 1(a)). QRT-PCR was performed to evaluate the H19 and miR-152 levels in the ox-LDL-treated HAECs. The results showed that compared with the control group, the expression of H19 in the ox-LDL group was significantly increased, but the expression of miR-152 was remarkably decreased (Figures 1(b) and 1(c), *P* < 0.05). This result indicates that H19 and miR-152 may involve the pathogenesis of the ox-LDL-induced atherosclerosis.

### 3.2. H19 Inhibited Cell Proliferation, Tube Formation, and Migration of the Ox-LDL-Induced HAECs

To further investigate the biological functions of H19 in the ox-LDL treated HAECs. We prepared H19 knockdown HAECs by H19 siRNA transfection. QRT-PCR analysis (Figure 2(a)) showed that compared with the siRNA scramble (si-NC) group, the expression of H19 in the H19 siRNA transfected (si-H19 group) HAECs were significantly downregulated. Further, compared with the siNC group, H19 knockdown significantly reduced cellular proliferation rate (Figure 2(b)), tube formation (Figure 2(c)), and cellular migration (Figure 2(d)) of the ox-LDL treated HAECs. E-cadherin and vimentin are reported to participate in the pathogenesis of atherosclerosis. Western blot detection indicated (Figure 2(e)) that compared with the siNC group, the E-cadherin protein expression in the si-H19 group cells was significantly increased, while vimentin expression was significantly reduced, indicating that knocking down H19 would reduce the epithelial-mesenchymal transformation (EMT) trend of the ox-LDL treated HAECs.

### 3.3. Expression of H19 Was Negatively Correlated to miR-152 in the Ox-LDL-HAECs

In order to study the molecular mechanism of H19, we determined whether H19 was expressed in the cytoplasm or the nucleus by qRT-PCR. The result showed that H19 was mainly expressed in the cytoplasm in the ox-LDL-HAECs (Figure 3(a)). Dual-luciferase experiment indicated that co-transfection of miR-152 mimics significantly inhibited the luciferase activity of the H19 vector (lncRNA H19-WT) but did not inhibit the luciferase activity of the lncRNA H19-MUT vector. Thus, the targeting relationship between H19 and miR-152 was confirmed (Figure 3(b)). In addition, compared with the siNC group, H19 knockdown significantly upregulated the expression of miR-152 (Figure 3(c)). The expression of H19 was negatively correlated to the miR-152 in the ox-LDL-HAECs (Figure 3(d)).

### 3.4. Knockdown of miR-152 Attenuated the si-H19 Induced Antiangiogenic Activities in the Ox-LDL-HAECs

Compared with the siNC + NC inhibitor group, the proangiogenic activity (including cellular proliferation rate, migration ability, tube formation ability, and EMT trend) of the si-H19 + NC inhibitor group cells was significantly reduced. On the contrary, the cellular proliferation rate, migration ability, tube formation ability, and EMT trend of the ox-LDL-HAECs increased significantly after interference with miR-152. Interestingly, miR-152 inhibitor transfection attenuated the antiangiogenic activity induced by si-H19 in the ox-LDL-HAECs (Figures 4(a)–4(d)).

### 3.5. VEGFA Is the Target Gene of miR-152, Which Is Regulated by H19 via miR-152

TargetScan database (http://www.targetscan.org/vert_72/) was applied to predict the target genes of miR-152. The prediction results show that there is a binding site between VEGFA and miR-152 (Figure 5(a)). Dual-luciferase assay was then applied to verify this prediction, which showed that miR-152 mimics significantly inhibited the luciferase activity of the VEGFA-WT carrier but did not inhibit the luciferase activity of the VEGFA-mutation (VEGFA-MUT) carrier (Figure 5(a)). These results confirmed the targeting relationship between miR-152 and VEGFA. To further verify this relationship, qRT-PCR and Western blot were performed and showed that compared with the NC mimics group, miR-152 mimics transfection significantly inhibited the expression of VEGFA mRNA and protein in the ox-LDL-HAECs (Figures 5(b)–5(c)). Correlation analysis revealed that miR-152 was negatively correlated with VEGFA (Figure 5(d)). In addition, compared with the siNC group, the expression of VEGFA in the ox-LDL-HAECs was significantly reduced after interference with si-H19, and the expression of H19 and VEGFA was positively correlated (Figures 5(e)–5(f)). At the same time, after interfering with the miR-152, the expression of VEGFA in the cells increased significantly. However, compared with the si-H19NC inhibitor group, miR-152 inhibitor can reverse the expression of VEGFA (Figures 5(g) and 5(h)).

### 3.6. Antiangiogenic Activity of miR-152 Inhibits via Downregulating VEGFA in the Ox-LDL-HAECs

The angiogenic assay was further applied to determine whether miR-152 could regulate HAECs by targeting VEGFA. Compared with the NC mimics + vector group, the proliferation rate (Figure 6(a)), migration ability (Figure 6(b)), tube formation ability (Figure 6(c)), and EMT trend (Figure 6(d)) of the ox-LDL-HAECs were significantly reduced after miR-152 mimic transfection. While these activities and EMT trend were significantly higher in the VEGFA overexpressed ox-LDL-HAECs. At the same time, overexpression of VEGFA can reverse the effect of miR-152 upregulation on the angiogenic activity of the ox-LDL-HACEs.

## 4. Discussion

Atherosclerosis is a chronic multifactorial vascular disease and the root cause of cardiovascular disease. It is characterized by lipid accumulation and the formation of fatty plaques in blood vessels [24]. Despite advances in treatment, the morbidity and mortality of atherosclerosis are still at a high level. Therefore, there is an urgent need to reveal detailed mechanism of atherosclerosis and find effective treatment targets and methods for atherosclerosis.

Studies have shown that ox-LDL has a bidirectional effect on angiogenesis [25]. Low concentrations of ox-LDL (less than 5 *μ*g/ml) stimulate VEGF expression, endothelial cell migration, and neocapillary formation [25, 26]. Therefore, in this study, 5 *μ*g/ml was used to induce HAECs into an atherosclerosis cell model. Previous studies have shown that expression of H19 is upregulated in cardiovascular diseases, including vascular smooth muscle cells [27]. This study also found that H19 was significantly upregulated in HAECs induced by 5 *μ*g/ml ox-LDL. Moreover, after knocking down the expression of H19, the proliferation, migration, and tube formation of ox-LDL-induced HAECs were significantly inhibited, which is similar to the role of the H19 in many cancer cells. For example, Zhao et al. found that knocking down H19 can significantly inhibit the proliferation and metastasis ability of lung cancer cell lines [28]. It is suggested that H19 has the potential to be a biomarker for diagnosing changes in the state of vascular endothelial cells, and H19 is related to the biological functions of cells.

According to previous research reports, lncRNA exhibits its activities in a variety of ways. It can participate in the regulation of protein before and after transcription to directly control the protein activity. It mainly includes direct binding to target protein to affect its function, or binding to miRNA or circRNA to participate in signal transduction and other ways [29]. Among them, miRNA is a type of short noncoding RNA with a length of about 22 nt [30]. Due to the high efficiency and specificity of miRNA, it is often used as a biomarker of disease [31]. Many studies have found that the expression of miR-152 is often downregulated in different solid tumors [32], suggesting that miR-152 can inhibit the biological activity of cancer, acting as a tumor suppressor. There have been some reports on the pathological regulation of the H19/miR-152 axis, which mostly involves cell proliferation, invasion, angiogenesis, and apoptosis. Li et al. [33] showed that in the study of diabetic foot ulcer repair, H19 inhibited the apoptosis and inflammation of fibroblasts by reducing the activity of miR-152-3p-mediated tensin protein homolog activity, thereby promoting wound healing of diabetic foot ulcers. In human glioma cells, the level of H19 increases, while the level of miR-152 decreases. Lowering H19 or increasing miR-152 can inhibit the proliferation and invasion of glioma cells to inhibit the growth of glioma cells [34]. The results of this study found that the expression of miR-152 was significantly downregulated in cardiovascular ox-LDL–treated HAECs. Dual-luciferase assay showed that H19 could bind miR-152. Knocking down H19 significantly upregulated miR-152 expression accompanied with antiangiogenic activity. Li et al. [35] showed that H19 can upregulate the expression of DNMT1 through sponge miR-152, thereby promoting the proliferation and invasion of breast cancer, suggesting that miR-152 is a key mediator for H19 to exert its biological functions. These data show that H19 has a negative regulatory effect on miR152. H19 is involved in the regulation of cell proliferation (vascular endothelial or tumor) through the negative regulation of miR152 to involve angiogenesis or tumor pathogenesis.

According to previous research reports, miRNA can bind to the 3′-UTR of a specific mRNA through its seed sequence to inhibit the translation of the mRNA and participate in the regulation of cell life activities [36]. This study also showed that miR-152 has a target relationship with VEGFA that is an important signal molecule leading to atherosclerosis. Balance of VEGFA is crucial to maintaining the physiological vascular homeostasis of cells and tissues [37]. High expression of VEGFA is the direct cause activating vascular endothelial cells. Haque et al. found that overexpression of miR-152 can significantly inhibit the expression of VEGF and TGF*β*1 in retinal endothelial cells [38]. Fu et al. [39] reported that overexpression of miR-152 can inhibit high glucose-induced angiogenesis in human retinal endothelium cells and retinal microvascular endothelial cell lines by targeting inhibition of VEGF signaling. All the data suggest that VEGF signal is the main target of miR-152 to inhibit angiogenesis.

## 5. Conclusion

In conclusion, H19 promotes cellular proliferation, migration, and angiogenesis through the miR-152/VEGFA axis in the ox-LDL-induced HAECs. These findings also suggested that H19 could be a target to regulate the biological activity of vascular endothelial cells. However, in order to reveal the relationship between ox-LDL and H19, further investigations are needed to more comprehensively elaborate the mechanism of ox-LDL causing changes in the activity of vascular endothelial cells.

## Figures and Tables

**Figure 1:** Ox-LDL induced upregulation of H19 expression and downregulation of miR-152 expression in ox-LDL-treated HAECs. A. Potential binding sites between miR-152 and lncRNA H19 (H19) were analyzed by DIANA-lncBase database. B. Expression of H19 was detected by qRT-PCR in the wild type HAECs (Control) and ox-LDL-treated HAECs. C. The expression of miR-152 was analyzed in the control and ox-LDL groups in HAECs. Each data were obtained from three different independent test results.  ^*∗∗*^*P* < 0.01.

**Figure 2:** Knockdown of H19 inhibited the ox-LDL-induced proangiogenic activities of HAECs. (a). Efficiency of the si-lncRNA H19 (si-H19) was evaluated by qRT-PCR in the ox-LDL-HAECs. (b). Cellular proliferation was detected by MTT in the indicated cells. (c) Tube formation was performed to detect the angiogenesis ability in the indicated cells. (d) Cellular migration was evaluated by Wound-healing assay in the indicated cells. (e) Protein expression of E-cadherin and vimentin was analyzed by Western blot.  ^*∗*^*P* < 0.05 and  ^*∗∗*^*P* < 0.01 *vs*. siNC group.

**Figure 3:** Expression of H19 was negatively correlated to the miR-152 in the ox-LDL-HAECs. (a) qRT-PCR detected the expression of H19 in the isolated cytoplasm and nucleus of the ox-LDL-HAECs.  ^*∗∗*^*P* < 0.01. (b) Binding relationship of the H19 and miR-152 were analyzed by Dual-luciferase assays.  ^*∗∗*^*P* < 0.01 *vs* mimics NC group. (c) qRT-PCR was used to detect the expression of miR-152 in the siNC group and si-H19 group in the ox-LDL-HAECs,  ^*∗∗*^*P* < 0.01. (d) Correlation between the expression of H19 and miR-152 was analysis by Pearson analyzes.

**Figure 4:** Low expression of miR-152 attenuated the si-H19-induced antiangiogenic activity in the ox-LDL-HAECs. Cellular proliferation, tube formation, migration, and protein expression of E-cadherin and vimentin were analyzed by MTT (a), Matrigel tuber formation (b), Wound-healing assay (c), and Western blot (d) in the ox-LDL-HAECs.  ^*∗∗*^*P* < 0.01 *vs* siNC + NC inhibitor group; ## *P* < 0.01 *vs* si-H19 + NC inhibitor group.

**Figure 5:** VEGFA is the target gene of miR-152, through which H19 can regulate the VEGFA expression. (a) Binding site between the miR-152 and VEGFA was predicated by TargetScan database analysis (up panel). Dual-luciferase analysis of miR-152 to VEGFA.  ^*∗∗*^*P* < 0.01 *vs* mimics NC. B–C. The expression of VEGFA mRNA and protein were analyzed by qRT-PCR (b) and Western blot (c) in the miR-152 mimics or mimics NC transfected ox-LDL-HAECs;  ^*∗∗*^*P* < 0.01. (d) Pearson analysis of the correlation between miR-152 and VEGFA expression. (e) VEGFA gene expression was detected by qRT-PCR in the si-H19 transfected ox-LDL-HAECs,  ^*∗∗*^*P* < 0.01. (f) Correlation of the expression of H19 and VEGFA was analyzed by Pearson analysis. **G-H**. VEGFA mRNA and protein expression were detected by qRT-PCR (g) and Western blot (h) in the indicated groups of the ox-LDL-HAECs.  ^*∗∗*^*P* < 0.01 *vs* siNC + NC inhibitor group, ## *P* < 0.01 *vs* si-H19 + NC inhibitor group.

**Figure 6:** Antiangiogenic activity of miR-152 by downregulating VEGFA in the ox-LDL-HAECs. Cellular proliferation (a), tube formation (b), wound-healing assay (c) were detected in the indicated groups. (d) E-cadherin and Vimentin protein levels were analyzed by Western blot.  ^*∗∗*^*P* < 0.01 *vs*. NC mimics + vector group, ## *P* < 0.01 *vs*. miR-152 mimics + vector group.

**Table 1:** qRT-PCR primers.

Target gene/RNA	Sequences (5′ to 3′)
lncRNA H19	F : ATCGGTGCCTCAGCGTTCGG
	R : CTGTCCTCGCCGTCACACCG

miR-152	F : CAGTGCATGACAGAACTTG
	R : GAACATGTCTGCGTATCTC

VEGFA	F : TTGCCTTGCTGCTCTACCTCCA
	R : GATGGCAGTAGCTGCGCTGATA

U6	F : ACCCGTTGAACCCCATTCGTGA
	R : GCCTCACTAAACCATCCAATCGG

GAPDH	F : CATCACTGCCACCCAGAAGACTG
	R : ATGCCAGTGAGCTTCCCGTTCAG

## Data Availability

The data used to support the findings of this study are available from the corresponding author upon request.
